The article "Clinical Observation of Flapless Implantation in the Posterior Tooth Area under the Guidance of the Fully Guided Template" was retracted in 2023. Reasons: signs of a paper mill; suspected computer-generated content; unreliable results or conclusions; concerns about the data.

# Clinical Observation of Flapless Implantation in the Posterior Tooth Area under the Guidance of the Fully Guided Template

**DOI:** 10.1155/2022/9270455

**Published:** 2022-07-06

**Authors:** Dan Wei, Weifeng Xu, Liangwu Chen, Hongyan Lu

**Affiliations:** Extraoral Implant Department, Ningbo Haishu Stomatological Hospital, Ningbo 315010, Zhejiang, China

## Abstract

**Objective:**

Compared with the conventional flap implantation, the postoperative effect of flapless implantation of a single posterior tooth under the guidance of the fully guided template was observed.

**Materials and Methods:**

67 cases were divided into the template group (*n* = 35) and the flap group (*n* = 32) according to the wishes and actual situation of the patients. In the template group, the fully guided template was made by rapid prototyping technology, and the flapless implantation was performed under the guidance of the template in the posterior tooth area. The flap group underwent routine flap implantation. After the operation, the template group took CBCT (cone beam computed tomography) again and fitted it with that before the operation. Neck deviation, apical deviation, depth deviation, and axial angle deviation in buccolingual and mesiodistal directions were measured to observe the accuracy of the fully guided template. At the same time, the postoperative reactions of the two surgical methods were compared by recording the operation time, pain degree 24 hours after the operation, swelling degree 72 hours after the operation, and postoperative satisfaction of patients.

**Results:**

Whether in buccolingual or mesiodistal directions, the maximum values of neck deviation, apical deviation, and depth deviation were less than 2 mm. The axial angle deviation was 0.07°∼5.93° in the buccolingual direction and 0°∼4.12° in the mesiodistal direction. The guiding effect of the template was relatively reliable, and the implantation site and depth were well controlled. Although there were small deviations, the accuracy of the template could meet the clinical needs. The operation time and the VAS (visual analogue scale) score 24 hours after the operation in the template group were lower than those in the flap group (*P* < 0.05), and the swelling degree rating 72 hours after the operation and postoperative satisfaction of the patients were better than those in the flap group (*P* < 0.05).

**Conclusion:**

Compared with the conventional flap implantation, the flapless implantation in the posterior tooth area under the guidance of the fully guided template could improve the accuracy of the operation, shorten the operation time, and reduce the degree of postoperative pain and swelling, which had a certain positive clinical significance.

The article "Clinical Observation of Flapless Implantation in the Posterior Tooth Area under the Guidance of the Fully Guided Template" was retracted in 2023. Reasons: signs of a paper mill; suspected computer-generated content; unreliable results or conclusions; concerns about the data.

## 1. Introduction

Traditional dental implant surgery needed to open the full-thickness flap of soft tissue and judge the bone mass and correct implant site under direct vision [1]. Although this operation method was conducive to reducing the operation risk, it was more traumatic and easy to swell after the operation, resulting in some patients unwilling to accept implant surgery. The emergence of the digital template provided a new auxiliary positioning method for implantation, making virtual planning predictable and accurate planting possible [2]. In particular, the fully guided template developed in recent years could guide the preparation of implant cavity and implantation process by replacing the sleeve. When the bone volume and keratinized gingiva in the operation area were sufficient, the circular cutting and minimally invasive implantation without flap turnover guided by the digital template could be performed to reduce the postoperative discomfort of patients. Compared with the conventional flap implantation, this paper observed the postoperative effect of flapless implantation of a single posterior tooth under the guidance of the fully guided template. It was evaluated from the two aspects, including the accuracy of the template and postoperative response, in order to provide reference for clinical practice.

## 2. Data and Methods

### 2.1. Materials and Equipment

3Shape TRIOS intraoral scanner (3Shape, Denmark), CBCT (Newton, Italy), Straumann BLT implant system, and full guide tool box (Straumann, Switzerland) were used in this study.

### 2.2. Case Data

This study was approved by the ethics committee of our hospital, and all subjects signed informed consent. 67 patients with single posterior tooth loss treated in our hospital from January 2021 to August 2021 were selected as the research object. Inclusion criteria: ① patients voluntarily required implant restoration and met the surgical indications and indications; ② CBCT examination and complete imaging data; ③ single posterior tooth was missing, and the implant area had sufficient bone mass and keratinized gingiva; ④ good oral hygiene. Exclusion criteria: ① patients with contraindications to implant; ② there were residual roots or granulation tissue in the implant area; ③ insufficient bone mass or keratinized gingiva in the implant area; ④ poor compliance or failure to follow-up and recheck as required. The patients were divided into the template group (*n* = 35) and the flap group (*n* = 32) according to their wishes and actual conditions. In the template group, there were 18 males and 17 females, aged 25–48 years, with 19 premolars and 16 molars. There were 17 males and 15 females in the flap group, aged 27–53 years, with 14 premolars and 18 molars.

The article "Clinical Observation of Flapless Implantation in the Posterior Tooth Area under the Guidance of the Fully Guided Template" was retracted in 2023. Reasons: signs of a paper mill; suspected computer-generated content; unreliable results or conclusions; concerns about the data.

### 2.3. Method

#### 2.3.1. Preoperative Preparation

Both groups underwent elective surgery. In the template group, CBCT and 3Shape TRIOS intraoral scanner were used to obtain the digital information of the implant area, respectively. After the two were integrated and matched on the computer, the position of the implant was preset on the software. After confirming the implantation scheme, the data such as the specification, direction, and depth of the implant were transformed into stereolithography format as parameters, and the fully guided template was made by rapid prototyping technology. CBCT was routinely taken in the flap group as a reference of the implant site and direction for the operator.

#### 2.3.2. Surgical Procedure

All operations were performed by implant doctors with certain clinical experience and good surgical ability. The patients were given oral antibiotics and mouthwash before the operation. Routine disinfection, towel laying, and local infiltration anesthesia were also carried out. Guided by the fully guided template, the template group performed minimally invasive implant surgery without flap turnover: put the preoperative soaked and sterilized template in place to ensure that the template was stable without looseness and in close contact with the remaining teeth. Straumann full guide tool box was used, changing the sleeve and corresponding reamer step by step according to the design requirements. Pay attention to cooling during the operation to prevent bone burns. Probe whether there was perforation of bone wall. After flushing the implant cavity with normal saline, the final forming drill and implant carrier were used to implant under the guidance of the fully guided template. The appropriate healing cap was selected without suture. In the flap group, the conventional flap fully exposed the alveolar bone in the implant area, expanded the hole step by step according to the predetermined implantation direction, implanted routinely, selected the appropriate healing cap, and finally sutured the wound tightly. In order to prevent infection, both groups were treated with oral antibiotics for 2 days.

### 2.4. Accuracy Evaluation of the Fully Guided Template

The patients in the template group took CBCT again after the operation and fitted it with that before the operation. The actual implant site and the virtual implant site were overlapped and matched [3]. The maximum axial sections of the implant in buccolingual direction and mesiodistal direction were intercepted on the three-dimensional images, and the centerline of the implant was extracted. The following four indexes were measured: ① neck deviation; ② apical deviation; ③ depth deviation; and ④ axial angle deviation (Figure 1).

The article "Clinical Observation of Flapless Implantation in the Posterior Tooth Area under the Guidance of the Fully Guided Template" was retracted in 2023. Reasons: signs of a paper mill; suspected computer-generated content; unreliable results or conclusions; concerns about the data.

### 2.5. Comparison of Operation-Related Indexes between the Two Groups

The following indexes of the two groups were recorded and compared. ① Operation time: the operation time of the two groups was recorded. ② Pain degree 24 hours after the operation: the visual analogue scale (VAS) was used, with a score of 0∼10. The higher the score, the more obvious the pain [4]. ③ Swelling degree 72 hours after the operation: it was mild if there was no obvious swelling in the implant area, or the swelling was limited within 2 mm around the abutment. It was moderate if the swelling was more than 2 mm around the abutment, but not more than the adjacent teeth. It was considered severe if the swelling was more than moderate. ④ Postoperative satisfaction: the postoperative satisfaction of patients was investigated and recorded, which was divided into very satisfied, generally satisfied, and dissatisfied.

### 2.6. Statistical Analysis

SPSS 19.0 statistical software was used for data analysis. The independent sample *t*-test or rank sum test should be adopted after the normality test of measurement data line. The rank sum test was used for rank data. When *P* < 0.05, the difference was statistically significant.

## 3. Results

### 3.1. Accuracy Evaluation of the Fully Guided Template

The measurement results of the four indexes in the template group are shown in Table 1. Whether in buccolingual direction or mesiodistal direction, the maximum values of neck deviation, apical deviation, and depth deviation were less than 2 mm. The axial angle deviation was 0.07°∼5.93° in the buccolingual direction and 0°∼4.12° in the mesiodistal direction. The guiding effect of the fully guided template was relatively reliable, and the implantation site and depth were well controlled. Although there were small deviations, the accuracy of the template could meet the clinical needs.

### 3.2. Comparison of Operation-Related Indexes between the Two Groups

Both groups of patients successfully completed the operation without serious complications, such as bone perforation and mandibular canal injury. The comparison results of operation related indexes are shown in Tables 2 and 3. The results showed that the differences of all indexes were statistically significant (*P* < 0.05). The operation time and the VAS score of pain 24 hours after the operation recorded in the template group were lower than those in the flap group, and the swelling degree rating 72 hours after the operation and postoperative satisfaction of patients were also better than those in the flap group.

The article "Clinical Observation of Flapless Implantation in the Posterior Tooth Area under the Guidance of the Fully Guided Template" was retracted in 2023. Reasons: signs of a paper mill; suspected computer-generated content; unreliable results or conclusions; concerns about the data.

## 4. Discussion

With the deepening of the concept of minimally invasive surgery, both doctors and patients hoped to complete the implantation operation through the smallest surgical incision and the least tissue trauma. Especially in the posterior tooth area, due to the small aesthetic impact, when the bone mass and keratinized gingiva were sufficient, the minimally invasive implantation of circumcision without flap turnover could be considered to simplify the operation and reduce the discomfort of patients. However, this technology required high experience of the operator. Because the operation was carried out under nondirect vision, the operator might misjudge the direction of the drill needle, resulting in poor implant placement and even lateral perforation of the bone plate. At the same time, because it was difficult to completely determine the thickness of the gum, it was difficult for the operator to control the implantation depth. With the continuous progress of the three-dimensional imaging technology and computer technology, the digital template was increasingly widely used in dental implant. By integrating the soft and hard tissue information obtained by CBCT and intraoral scanning, the digital template could transfer the implantation site, direction, angle, and depth preset on the computer to the practical operation [5] and help doctors find the best implantation site. It realized the perfect combination of minimally invasive technology and digital technology [6]. Especially under the guidance of the fully guided template, the operator could fix and expand the implant site by replacing the sleeve step by step and effectively prevent the drill needle from sliding. It could reduce the horizontal displacement of the final implant site. At the same time, the implant carrier in the tool box could also be used to complete the final implant under the guidance of the template, and the control of depth was more ideal.

In the process of using the digital template, its accuracy was an important factor affecting the success of planting. Many studies had shown that the application of the digital template could improve the accuracy of implant surgery compared with free-handed implantation [7], and most scholars believed that the full guidance was better than partial guidance in terms of accuracy [8, 9]. However, it was difficult to completely avoid the error in the process of design, manufacture, and practical application of the digital template, so there was still a certain deviation between the actual implant site and the virtual site designed before the operation. This was the result of error accumulation in the whole digital workflow [10]. Many similar studies and reports set 2 mm as the safe distance for the application of the digital template [11, 12]. In this study, the axial angle deviation was 0.07°∼5.93° in the buccolingual direction and 0°∼4.12° in the mesiodistal direction, indicating that the guidance of the fully guided template was relatively reliable and the drill needle was not easy to offset. No matter in the buccolingual direction or mesiodistal direction, the maximum values of neck deviation, apical deviation and depth deviation of the implant in the template group were less than 2 mm safe distance, especially depth deviation, which was 0.05 mm∼0.77 mm in the buccolingual direction and 0.02 mm∼0.72 mm in the mesiodistal direction. It showed that the fully guided template could improve the accuracy of flapless implant surgery. Under the guidance of the template, the implantation site and depth were well controlled. The implantation accuracy was high, although there was a small deviation, but its safety could meet the clinical requirements. However, it was worth noting that the flapless implantation was carried out under blind vision, which increased the uncertainty of surgical operation. Therefore, it was necessary to select cases with sufficient bone mass when applying the template. The error of the template should also be fully considered. It was recommended to leave sufficient safety distance so as not to damage important anatomical structures such as the mandibular canal [13]. At the same time, it was necessary to ensure the accuracy and stability of the template in place during the operation, and the operator should perform the operation according to the procedures. The template could not be completely relied on during the operation. Careful exploration was needed before the implantation to clarify the integrity of the bone plate.

The article "Clinical Observation of Flapless Implantation in the Posterior Tooth Area under the Guidance of the Fully Guided Template" was retracted in 2023. Reasons: signs of a paper mill; suspected computer-generated content; unreliable results or conclusions; concerns about the data.

As for the operation time and the postoperative response, some studies indicated that the flapless procedure showed advantages in preserving the gingival papilla, reducing postoperative pain and peri-implant probing depth compared to the flap procedure. Therefore, the flapless technique was more recommended in the ideal implantation site of soft and hard tissue [14]. The results of this study showed that the operation time and the VAS score of pain 24 hours after the operation in the template group were lower than that in the flap group (*P* < 0.05), and the swelling degree rating 72 hours after the operation and postoperative satisfaction were better than that in the flap group (*P* < 0.05). When the operation was performed under the guidance of the fully guided template, the implantation site, direction, and depth of the implant were planned before the operation. The operator could complete the operation under the guidance of specific tools, and there was no need for suture after the operation. The wound could be filled by directly placing a suitable healing cap, which effectively shortened the operation time. At the same time, because there was no need to turn over the flap to peel off the periosteum, the surgical trauma was small. The shape of gingival papilla and blood supply were preserved as much as possible, which was conducive to the health of soft and hard tissues in the implant area. After removing the gums by circumcision and placing the healing cap, the surrounding gums would not be pulled or compressed, which was conducive to the formation of epithelial cuff closure and effectively isolate the oral bacterial environment. Therefore, the patients in the template group recovered better. They had less bleeding and infection and less pain and swelling than the conventional flap group, and their satisfaction was also higher.

In conclusion, it provided a good method to use the minimally invasive implantation without flap turnover in the posterior tooth area under the guidance of the fully guided template. The template could guide the implant into the preset site before the operation more accurately. In this way, human errors could be reduced, the operation time could be shortened, postoperative pain and swelling could be eased, and patients may have a high degree of satisfaction, which had a certain positive clinical significance. However, doctors should pay attention to the selection of indications and strictly control various details to improve the success of implant surgery.

## Figures and Tables

**Figure 1:** The diagram of four measurement indexes.

**Table 1:** Measurement results of four indexes of the template group (*n* = 35).

Statistic	Buccolingual direction				Mesiodistal direction			
	Neck deviation (mm)	Apical deviation (mm)	Depth deviation (mm)	Axial angle deviation (°)	Neck deviation (mm)	Apical deviation (mm)	Depth deviation (mm)	Axial angle deviation (°)
Minimum	0.18	0.21	0.05	0.07	0.09	0.09	0.02	0.00
Maximum	1.57	1.62	0.77	5.93	1.42	1.57	0.72	4.12
Mean	0.80	0.92	0.42	1.76	0.82	0.84	0.40	1.70
Std. deviation	0.40	0.43	0.22	1.26	0.40	0.45	0.20	1.20

**Table 2:** Comparison of the operation time and the VAS score of pain 24 hours after the operation between the two groups.

	Operation time (min, ±s)	VAS score of pain 24 hours after the operation (score, ±s)
The template group (*n* = 35)	23.63 ± 3.07	2.46 ± 0.98
The flap group (*n* = 32)	29.78 ± 3.34	3.38 ± 1.07
*t/Z*	*t* = −7.861	*Z* = −3.290
*P*	*P* < 0.05	*P* < 0.05

*Note*. Operation time: the data of the two groups conformed to the normal distribution, and the independent sample *t*-test was used; VAS score of pain 24 hours after the operation: the data did not conform to the normal distribution, and the rank sum test was used.

The article "Clinical Observation of Flapless Implantation in the Posterior Tooth Area under the Guidance of the Fully Guided Template" was retracted in 2023. Reasons: signs of a paper mill; suspected computer-generated content; unreliable results or conclusions; concerns about the data.

**Table 3:** Comparison of the swelling degree 72 hours after the operation and the postoperative satisfaction between the two groups.

	Swelling degree 72 hours after the operation (*n* (%))			Postoperative satisfaction (*n* (%))		
	Mild	Moderate	Severe	Very satisfied	Generally satisfied	Dissatisfied
The template group (*n* = 35)	27 (77.14%)	8 (22.86%)	0 (0%)	22 (62.86)	13 (37.14%)	0 (0%)
The flap group (*n* = 32)	16 (50%)	16 (50%)	0 (0%)	12 (37.5%)	20 (62.5%)	0 (0%)
*Z*	−2.297			−2.058		
*P*	*P* < 0.05			*P* < 0.05		

*Note*. The rank sum test was used for grade data.

## Data Availability

The data used to support the findings of this study are available from the corresponding author upon request.
